# Application Effect and Evaluation of Two-Dimensional Speckle Tracking Imaging on Myocardial Damage in Patients with Malignant Lymphoma Treated with Anthracyclines

This article has been retracted.

**DOI:** 10.1155/2021/6355047

**Published:** 2021-10-19

**Authors:** Chunqiang Bai, Fanyue Meng, Peiming Feng, Wan Wang, Liang Fang, Qiankun Chang, Lihong Wang

**Affiliations:** ^1^Department of Ultrasonography, The Affiliated Hospital of Chengde Medical College, Chengde 067000, China; ^2^Department of MEC Ultrasound, Chengde Center Hospital, The Second Affiliated to Chengde Medical University, Chengde 067000, China; ^3^Department of Hematology, The Affiliated Hospital of Chengde Medical College, Chengde 067000, China

## Abstract

**Objective:**

The purpose was to study the monitoring effect and application value of two-dimensional speckle tracking imaging (2D-STI) on myocardial function in patients with malignant lymphoma after treatment with anthracyclines.

**Methods:**

50 patients with malignant lymphoma treated in our hospital from June 2017 to December 2019 were randomly selected and were treated with anthracyclines to compare the cardiac global longitudinal strain (GLS), global radial strain (GRS), global circumferential strain (GCS), left ventricular twist (LVtw), GLS × LVtw, and changes of atrioventricular inner diameters before and after 3 cycles of treatment. According to the pathological examination results, the accuracy of 2D-STI in the detection of changes in myocardial function of patients was also clarified.

**Results:**

The absolute values of GLS, GRS and GCS after treatment were significantly lower than those before treatment, with statistical significance (*P* < 0.05). The LVtw and GLS × LVtw after 3 cycles of treatment were significantly lower than those before treatment, with statistical significance (*P* < 0.05). There was no significant difference in the atrioventricular inner diameters of patients before and after treatment, with no statistical significance (*P* > 0.05). There was no significant difference between the monitoring results of 2D-STI and the pathological examination results, with no statistical significance (*P* > 0.05).

**Conclusion:**

Anthracyclines can cause some myocardial damage in patients with malignant lymphoma. The application of 2D-STI to monitor the changes in myocardial function of patients can give more accurate monitoring results, facilitating the early implementation of appropriate treatment.

## 1. Introduction

As a common malignant tumor with high mortality and high recurrence rate, malignant lymphoma mainly occurs in lymph nodes or lymphatic tissue outside lymph nodes, and patients with malignant lymphoma need timely treatment after diagnosis [1–3]. At present, chemotherapy is commonly used in clinical treatment in which drugs are used to control the spread of tumor cells and inactivate tumor cells. However, chemotherapy drugs also have certain effects on other parts of the human body or body function when playing an antitumor role [4–6]. Many studies have reported that chemotherapy has certain damage to the human body, and the current research direction of relevant clinical medicine is to reduce the damage caused by chemotherapy to the human body [7–9]. As chemotherapeutic drugs with the main function of antitumor effect, anthracyclines are widely used in treating various types of solid tumors and hematological tumors. However, clinical trials have shown that anthracyclines can cause severe damage to the heart of patients during use and impair myocardial function and myocardial cell activity, leading to serious heart disease in patients [10, 11]. Electrocardiogram, ultrasound, MRI, and blood index examination are commonly used in the diagnosis and detection of myocardial damage caused by anthracyclines. However, the abovementioned examination methods are not sensitive to slight myocardial damage and may often ignore relatively slight myocardial damage, resulting in misdiagnosis and missed diagnosis. Two-dimensional speckle tracking imaging (2D-STI) is a newly developed ultrasonic technology. It utilizes the original acoustic speckle marks of myocardium to accurately track the movement of target myocardial tissue at continuous frame rate, detects the motion trace of the speckle in the whole cardiac cycle from the frame-by-frame tracking mark, and obtains the myocardial mechanical parameters such as speed, displacement, strain, strain rate, and torsion angle of myocardial tissue movement, to evaluate the overall and local function of the myocardium. It has been applied to evaluate the cardiac function of many heart diseases and is more sensitive than conventional ultrasound examination. It has also been used for the detection of cardiotoxicity induced by chemotherapy drugs and for the development of advanced cardiotoxicity prediction studies. In this study, patients with malignant lymphoma treated with anthracyclines were selected as research subjects to analyze the application value of 2D-STI in detecting the degree of myocardial damage in patients, specifically reported as follows.

## 2. Materials and Methods

### 2.1. General Information

50 patients with malignant lymphoma treated in our hospital from June 2017 to December 2019 were randomly selected, including 21 males and 29 females. They were aged 39–67 years, with an average age of (51.22 ± 3.39) years, an average course of (6.00 ± 1.34) months, an average height of (166.29 ± 10.30) cm, and an average weight of (70.38 ± 5.91) kg. There were 8 patients with diabetes mellitus, 11 patients with hypertension, and 4 patients with hyperlipidemia. There were 35 patients of diffuse large B-cell lymphoma (DLBCL), 8 patients of follicular lymphoma (FL), 4 cases of mantle cell lymphoma (MCL), 2 patients of marginal lymph node B-cell lymphoma (NMZL), and 1 patient of peripheral T-cell lymphoma (PTCL). There were 8 patients in stage II, 16 patients in stage III, and 26 patients in stage IV.

### 2.2. Inclusion/Exclusion Criteria

#### 2.2.1. Inclusion Criteria

1. The patients were consistent with the clinical manifestations of malignant lymphoma
2. The patients were between 18 and 70 years
3. The patients had no other organic diseases with normal renal function
4. The patients had no history of drug allergy or drug abuse and had no bad habits
5. The study was approved by the hospital ethics committee, and the patients voluntarily participated in the study and signed the informed consent

### 2.3. Exclusion Criteria

1. The patients had other tumors
2. The patients had a heart disease history and arrhythmia
3. The patients had consciousness disorder and did not cooperate with the research

### 2.4. Methods

All patients received chemotherapy with anthracyclines, for 21 days as one cycle. 2D-STI was used to detect the myocardial function of the patients before and after 3 cycles of chemotherapy, respectively, and to observe whether there was myocardial damage during treatment. The 2D-STI examination was performed by the same group of high-calibre ultrasound doctors using the same ultrasound diagnostic apparatus. The Philips digital high-grade cardiac color Doppler ultrasound diagnostic apparatus (manufacturer: Jiangsu Anmao Medical Technology Co., Ltd.; Batch No.: SFDA Certified No. 20152221796; Model: EPIQ7C) was used for detection, with the probe frequency of 3.0–7.0 MHz. The probe was placed on the front chest of the patient and moved to scan the heart of the patient to observe the changes in myocardial function. Clear views of the four-chamber, two-chamber, and three-chamber views of the left ventricular apex, as well as the levels of the short-axis mitral valve and papillary muscle of the parasternal great artery and the horizontal view near the apex, were acquired and stored for three consecutive cardiac cycles. The cardiac global longitudinal strain (GLS), global radial strain (GRS), global circumferential strain (GCS), left ventricular twist (LVtw), GLS × LVtw, and changes of atrioventricular inner diameters were monitored, and the myocardial indexes after 3 cycles of treatment were compared with those before treatment, aiming to analyze the effect of anthracyclines on the myocardium of patients with malignant lymphoma [12–14].

### 2.5. Observation Indexes

The cardiac GLS, GRS, GCS, LVtw, and GLS × LVtw and changes of atrioventricular inner diameters were compared before and after 3 cycles of treatment. According to the pathological examination results, the accuracy of 2D-STI in the detection of changes in myocardial function of patients was also clarified.

QLAB software was used to detect and analyze the cardiac GLS, GRS, GCS, LVtw, and GLS × LVtw. The atrioventricular inner diameters were directly reflected in the 2D-STI results, and the accuracy of 2D-STI was obtained after the 2D-STI results were compared with the pathological examination results.

### 2.6. Statistical Treatment

In this study, SPSS20.0 was the data processing software, and GraphPad Prism 7 (GraphPad Software, San Diego, USA) was used to draw pictures of the data. The study included count data and measurement data. The measurement data were measured by the *t*-test, expressed by ($\bar{\text{x}}$ ± *s*), and the count data were tested by *X*^2^, expressed by [*n* (%)]. The difference was statistically significant when *P* < 0.05.

## 3. Results

### 3.1. Comparison of GLS, GRS, GCS, and LVtw before and after Treatment

The absolute values of GLS, GRS, and GCS after 3 cycles of treatment were significantly lower than those before treatment, with statistical significance (*P* < 0.05). The LVtw of patients after 3 cycles of treatment was significantly lower than that before treatment, with statistical significance (*P* < 0.05), as shown in Figures 1–5.

### 3.2. Comparison of Atrioventricular Inner Diameters before and after Treatment

There was no significant difference in the atrioventricular inner diameters of patients before and after treatment (*P* > 0.05), as shown in Table 1.

### 3.3. Comparison of GLS × LVtw before and after Treatment

The GLS × LVtw of patients after 3 cycles of treatment was significantly lower than that before treatment (*P* < 0.05), as shown in Figure 6.

### 3.4. Accuracy of 2D-STI

All the patients showed myocardial damage after treatment with anthracyclines, and the pathological examination result was 100%. By comparison, the results showed that there was no significant difference between the 2D-STI detection results and the pathological examination results (*P* > 0.05), as shown in Table 2.

## 4. Discussion

Cancer patients need chemotherapy or radiotherapy to prolong life and control the development and spread of tumor cells in the body. However, radiotherapy and chemotherapy may have an impact on other body functions of patient, especially for skin, heart, lung, and renal function [15–17]. Therefore, patients treated with chemoradiotherapy often take drugs to protect organs and reduce the impact of chemoradiotherapy on other organ functions. Anthracyclines are commonly used chemotherapeutic drugs in clinic, which play a significant role in the treatment and control of various visible tumors and hematological tumors, with excellent treatment results [18–20]. However, clinical trials have shown that anthracyclines have a great impact on myocardial function of patients, and chemotherapy with anthracyclines may cause myocardial damage in patients. Generally speaking, ultrasonic diagnosis is a common diagnostic method for patients with myocardial damage, but it is not prominent in terms of detection rate and has the disadvantages of invasive examination, radioactive damage, low resource allocation and specificity, etc. Routine echocardiography is the most commonly used monitoring tool, but abnormalities or morphological changes in LVEF occur only when the myocardium is severely damaged or the heart as a whole is damaged. Therefore, LVEF is not a sensitive indicator for monitoring subclinical cardiotoxicity.

The expert consensus of the American Echocardiography Society emphasizes the applicability of 2D-STI to monitor early subclinical left ventricular systolic dysfunction associated with cancer treatment, suggesting that its parameters may enable accurate stratification of cardiac risk and facilitate timely intervention. Not only longitudinal and circumferential displacement but also torsional movement occurs during myocardial contraction. GLS, GRS, and GCS are the main parameters for 2D-STI to detect myocardial strain. LVtw is also a sensitive parameter for the evaluation of cardiac subclinical damage. The LVtw is mainly generated due to the movement of myocardial spiral myofibers, which are distributed in the endocardium and epicardium, with opposite directions. When the heart contracts, the apex of the heart rotates in the opposite direction from the base of the heart, and the sum of the rotation angles is the LVtw. The results of this study showed that the absolute values of GLS, GRS and GCS, and LVtw and GLS × LVtw in patients after 3 cycles of treatment with anthracyclines were significantly lower than those before treatment. There was no significant difference in the atrioventricular inner diameters of patients before and after treatment, which was mainly because of the short time of chemotherapy (3 cycles of treatment). Zhang Fan et al. [21] stated in their study that anthracyclines have a great impact on the myocardial function of patients with malignant lymphoma, but will not cause significant changes in cardiac structure in the short term, which is consistent with the conclusion of this study and fully proves the scientificity and reliability of the results of this study.

2D-STI is a new ultrasonic diagnostic technique. It has been reported that 2D-STI has better effect in myocardial diagnosis than ordinary ultrasonic diagnosis [22–25]. In order to study the effect of anthracyclines on the myocardium of patients with malignant lymphoma and the application value of 2D-STI in myocardial diagnosis, this study took patients with malignant lymphoma treated with anthracyclines as research subjects, compared the changes in myocardial function before and after treatment, and compared the 2D-STI detection results with the pathological examination results to analyze the application value of 2D-STI. 2D-STI was used to diagnose myocardial function, and the results showed that the accuracy of 2D-STI was 98%, which was not significantly different from that of pathological examination results (*P* > 0.05). This indicates that 2D-STI has high application value in the diagnosis of myocardial damage in patients with malignant lymphoma, which is worthy of clinical promotion and application.

In conclusion, anthracyclines can cause some myocardial damage in patients with malignant lymphoma and 2D-STI can accurately diagnose the degree of myocardial damage. Therefore, 2D-STI has high application value in clinic, which is worthy of promotion and application.

## Figures and Tables

**Figure 1:** Comparison of GLS and GCS before and after treatment. The abscissa from left to right represents GLS and GCS, and the ordinate represents the detection data (%). *∗* indicates the comparison of GLS before treatment (−20.66 ± 3.59%) and after 3 cycles of treatment (−15.62 ± 2.24%), with statistical significance (*t* = 8.422, *P* < 0.001). *∗∗* indicates the comparison of GCS before treatment (−18.29 ± 3.37%) and after 3 cycles of treatment (−14.08 ± 2.00%), with statistical significance (*t* = 7.597, *P* < 0.001).

**Figure 2:** Comparison of GRS before and after treatment. The abscissa from left to right represents before treatment and after 3 cycles of treatment, and the ordinate represents the GRS detection result (%). *∗* indicates the comparison of GRS before treatment (22.05 ± 5.56%) and after 3 cycles of treatment (17.63 ± 4.29%), with statistical significance (*t* = 4.450, *P* < 0.001).

**Figure 3:** Comparison of LVtw before and after treatment. The abscissa from left to right represents before treatment and after 3 cycles of treatment, and the ordinate represents the LVtw detection result (°). *∗* indicates the comparison of LVtw before treatment (9.56 ± 1.25°) and after 3 cycles of treatment (5.68 ± 0.89°), with statistical significance (*t* = 17.880, *P* < 0.001).

**Figure 4:** 2D-STI images of patients before treatment, LVEF before treatment (55.5%), GLS before treatment (−21.2%), GCS before treatment (−17.5%), GRS before treatment (23.8%), and LVtw before treatment (9.7°).

**Figure 5:** 2D-STI images of patients after 3 cycles of treatment. After 3 cycles of treatment, the myocardial strain decreased significantly, LVEF after 3 cycles of treatment (32.9%), GLS after 3 cycles of treatment (−15.0%), GCS after 3 cycles of treatment (−14.1%), GRS after 3 cycles of treatment (17.8%), and LVtw after 3 cycles of treatment (5.8°).

**Figure 6:** Comparison of GLS × LVtw before and after treatment. The abscissa from left to right represents before treatment and after 3 cycles of treatment, and the ordinate represents the GLS × LVtw detection result. *∗* indicates the comparison of GLS × LVtw before treatment (−168.52 ± 40.21) and after 3 cycles of treatment (−89.63 ± 33.67), with statistical significance (*t* = 10.650, *P* < 0.001).

**Table 1:** Comparison of changes in atrioventricular inner diameters of patients ($\bar{\text{x}}$ ± *s*, mm).

Time	Left atrial diameter	Left ventricular dimension	Right atrial diameter	Right ventricle dimension
Before treatment	31.05 ± 5.61	42.33 ± 5.06	30.29 ± 3.66	21.88 ± 3.01
After 3 cycles of treatment	31.66 ± 5.38	42.91 ± 5.19	30.58 ± 3.19	21.47 ± 3.48
*t*	0.554	0.566	0.422	0.630
*P*	0.580	0.573	0.674	0.530

**Table 2:** Accuracy of 2D-STI.

Group	Before treatment	After 3 cycles of treatment (%)
2D-STI	0%	98
Pathological examination	0%	100
*X* ^2^	1.014	
*P*	0.327	

## Data Availability

The primary data to support the results of this study are available at reasonable request to the corresponding author.
